This article has been retracted.

# Effects of Dexmedetomidine on Hemodynamics and Anesthesia Effect of Different Doses of General Anesthesia in Patients Undergoing Hepatobiliary Surgery

**DOI:** 10.1155/2022/2311869

**Published:** 2022-07-19

**Authors:** Zhaolong He, Jianan Du, Xiaolu Xue, Liu Yang

**Affiliations:** ^1^Department of Anesthesiology, The People's Hospital of Kizilsuch Kirghiz Autonodour Prefecture, Xinjiang 845350, China; ^2^Department of Anesthesiology, Sanya Central Hospital, Hainan Third People's Hospital, Sanya 572000, China; ^3^Department of Anesthesiology, The Second Affiliated Hospital of Kunming Medical University, Kunmings 650000, China

## Abstract

In order to provide corresponding anesthesia methods of hepatobiliary diseases and obtain better clinical effect, the hemodynamics and clinical efficacy are evaluated by using different doses of dexamethasone (DEX) during the operation. 97 patients undergoing general anesthesia for hepatobiliary surgery in our hospital from April 2020 to August 2021 are analyzed retrospectively. All patients are divided into G1 (*n* = 24), G2 (*n* = 24), G3 (*n* = 24), and control group (*n* = 25) according to the random number table method. The G1, G2, and G3 groups are injected with DEX 1.0 ug/kg, DEX 0.8 ug/kg, and DEX 0.5 ug/kg by intravenous infusion pump before induction of general anesthesia, and the control group is injected with 0.9%Nacl solution 10 mL. Intraoperative anesthesia time, postoperative eye opening time, and extubation time of all groups are observed, and the incidences of postoperative adverse reactions are compared. The experimental results show that during general anesthesia in the liver and gallbladder surgery, the patients with high dose of DEX can better maintain the intraoperative hemodynamic parameters, and effectively restrain the postoperative stress reaction.

## 1. Introduction

As an important organ of human body, liver and gall can regulate digestion, blood transport, and other physiological functions [1]. However, with the continuous improvement of social and economic level and the change of diet structure, the incidence rate of cholecystitis, hepatitis, liver cirrhosis, fatty liver, and other hepatobiliary diseases is also increasing [2]. Hepatobiliary surgery is an upper abdominal surgery with large trauma area. Due to the large tissue trauma involved, the time of hepatobiliary surgery is relatively long, and adverse events such as liver injury often occur during the operation [3]. Therefore, the operation of hepatobiliary diseases requires high anesthesia. Some studies have pointed out that anesthesia, as the basis for smooth operation, also has an important impact on the curative effect. Dexmedetomidine (DEX), as a receptor agonist, has a high analgesic effect in clinical practice [4].

Dexmedetomidine is *α*2 receptor agonists, and *α*2 exists in the anterior membrane of the synapse. By exciting *α*2 receptor, it can inhibit the release of catecholamines from the anterior neural membrane [5, 6]. Dexmedetomidine injection is usually used in general anesthesia, mechanical ventilation, and endotracheal intubation to make patients more stable during general anesthesia, surgery, or treatment. If intravenous injection or intravenous drip is carried out, the speed of reaching the peak will be accelerated, and it is usually excreted through the kidney. For critically ill patients under intensive care and treatment, patients need general anesthesia before operation, and then need tracheal intubation and mechanical ventilation [7]. At this point, dexmedetomidine is required to play a good sedative role to help doctors and patients with the next step of treatment. Dexamethasone, like other glucocorticoids, has the pharmacological effects of anti-inflammatory, anti-endotoxin, inhibiting immunity, antishock, and enhancing stress response. It can be used to treat acute severe bacterial infection, severe allergic diseases, purpura caused by various thrombocytopenia, granulocytopenia, as well as various serious skin diseases, immune rejection of organ transplantation. To some extent, dexamethasone is also an anti-inflammatory drug, which inhibits the growth of inflammatory cells, engulfs macrophages and leukocytes, and dissipates inflammation. Although dexamethasone plays an important role in the clinical efficacy of hepatobiliary general anesthesia, the specific effects of different doses of dexamethasone on patients undergoing general anesthesia have not been reported in most studies [8, 9].

This paper is organized as follows: Section 2 discusses the related work, and Section 3 presents the proposed methods and observation indicators. In Section 4, the comparative results and analysis is proposed. Finally, in Section 5, some concluding remarks are made.

## 2. Related Work

Relevant studies at home and abroad have shown that dexamethasone, as a highly selective adrenergic receptor agonist, can dilate blood vessels by stimulating vascular endothelial cells and sympathetic presynaptic membrane receptors [10]. Therefore, it can also be used in clinical practice to reduce the body pressure caused by endotracheal intubation [11, 12]. With the increase of DEX dose, the hemodynamic parameters will be more stable. This is because DEX plays an important role in stabilizing the dimensionality of patients. However, since DEX can be activated *α* 2-adrenaline, patients can also show the clinical phenomenon of elevated blood pressure in a short time [13, 14]. In addition, some scholars have shown that the speed of DEX administration will also have an impact on hemodynamic parameters, and excessive help speed will lead to hypertension symptoms. Further research is needed in this regard [15]. In addition, the effect of DEX on stress response should be considered. As hepatobiliary surgery is a major traumatic operation, the pain during operation and operation will stimulate a large number of stress factors in the body, thus secreting more prostacyclin. Sympathetic nerves secrete a lot of Cor, E, and NE after being stimulated by trauma [16]. The above indicators can be tested to reflect the stress state of patients. Some studies have shown that the stress response of patients decreases with the increase of DEX dose, further indicating that high-dose DEX plays an important role in reducing the posttraumatic stress response of patients [17].

The dose of DEX may affect the anesthesia time, the postoperative eye-opening time, and the extubation time [18, 19]. It is further suggested that DEX has a highly selective excitatory effect on *α*2 adrenalin receptors in the locus coeruleus of the brain and can effectively inhibit the discharge function of neurons, thus exerting analgesic and sedative effects. Therefore, increasing the amount of DEX during surgery can significantly prolong the anesthesia time and effect [20, 21]. However, at the same time, high-dose DEX over inhibited neurons in the brain, resulting in a corresponding increase in subsequent eye opening time. In contrast, according to the results of postoperative complications, the increase of intraoperative DEX dose will significantly increase the incidence of postoperative complications. Therefore, we do not blindly pursue high-dose DEX [22–24] during clinical anesthesia surgery.

In the courage process of general surgery, the use of high-dose DEX can effectively maintain the stability of perioperative hemodynamic parameters and reduce postoperative stress response to a certain extent [25]. However, high-dose DEX over inhibited the receptor will result in prolonged awakening time and increased incidence of postoperative complications [26]. In clinical anesthesia surgery, the appropriate DEX dose can be selected according to the patients' different physical qualities and personal conditions to further reduce postoperative complications on the premise of ensuring the anesthesia effect.

## 3. Proposed Methods and Observation Indicators

A retrospective analysis is performed on 97 patients undergoing hepatobiliary surgery under general anesthesia in our hospital from April 2020 to August 2021. All patients are divided into G1 (*n* = 24), G2 (*n* = 24), G3 (*n* = 24), and control group (*n* = 25) according to the random number table method. The G1, G2, and G3 groups are injected with DEX 1.0 ug/kg, DEX 0.8 ug/kg, and DEX 0.5 ug/kg by intravenous infusion pump before induction of general anesthesia, and the control group is injected with 0.9%Nacl solution 10 mL. The comparison of baseline data of each group is shown in Table 1, which is comparable (*P* > 0.05). All patients included in the study signed informed consent before surgery and obtained the right to know and consent to all operations during surgery. The clinical data and general information obtained in this study are kept confidential and will not be used for other purposes.

Inclusion criteria are as follows: (1) patients with surgical indications; (2) sign preoperative informed consent; (3) complete clinical data and general information; and (4) ASA classification is I∼II. Exclusion criteria are as follows: (1) patients with a history of allergy to intraoperative anesthetic drugs; (2) people with coagulation disorder; (3) complicated with heart, liver, kidney, and other major organ diseases; and (4) patients with mental diseases cannot communicate effectively with researchers. Table 1 shows the baseline data.

### 3.1. Method of Anesthesia

Before surgery, all patients underwent general physical examination, fasting, and water prohibition for 12 hours. After entering the operating room, patients in 4 groups underwent routine electrocardiogram, arterial pressure, heart rate, and blood oxygen saturation detection and established venous channels. In G1, G2, and G3 groups, 1.0 ug/kg, DEX 0.8 ug/kg, and DEX 0.5 ug/kg are pumped at constant speed 15 min before anesthesia induction, while in the control group, 10 mL of 0.9% NaCl solution is injected. Dex0.5 ug and 0.02 ug sufentanil are pumped continuously until 15 min before the end of surgery. Tracheal intubation and mechanical ventilation are performed after anesthesia induction, tidal volume 8–10 mL/kg, frequency 10–12 times/min. After surgery, the patient is sent to the recovery room for real-time monitoring of vital signs and assisted breathing according to personal conditions.

Plasma cortisol (Cor), epinephrine (E), and norepinephrine (NE) are detected by radioimmunoassay before and after operation in 4 groups.

### 3.2. Observation Indicators

The observation indicators are as follows: (1) The changes of hemodynamic parameters at T1, T2, T3, and T4 time points are recorded; (2) Cor, E, and NE levels are observed before and after surgery; (3) intraoperative anesthesia time, postoperative eye opening time, and extubation time are observed in each group; and (4) the incidence of postoperative adverse reactions is observed.

SPSS 25.0 statistical software is used for data analysis, and the specific steps are as follows: (1) Measurement data: If the data followed normal distribution and homogeneity of variance after normality test, they are represented by mean ± standard deviation. Paired sample *T* is used for intragroup test, and variance comparison is used between groups. Repeated measurement ANOVA is used for spherical test at each time between groups. (2) Count data: Descriptive statistical analysis is conducted by percentage, and *χ*^2^ test is performed. *P* < 0.05 indicated significant difference.

## 4. Results and Analysis

### 4.1. Comparison of the Changes of Hemodynamic Parameters in T1, T2, T3, and T4

Heart rate changes in each group are shown in Table 2 and Figure 1. Systolic blood pressure is shown in Table 3 and Figure 2. The symbol “*∗*” means that compared with G1, *∗P* < 0.05. The symbol “#” indicates that compared with G2, #*P* < 0.05. The symbol “&” means compared with G3, &#*P* < 0.05. Besides, the symbol “a” means that compared with T1, a*P* < 0.05. The symbol “b” means that compared with T2, b*P* < 0.05, and the symbol “c” means that compared with T3, c*P* < 0.05. The diastolic pressure changes are shown in Table 4 and Figure 3. The results indicate that compared with G2, G3, and the control group, G1 has the most stable hemodynamic parameters during the whole surgical process and can maintain similar hemodynamics after extubation as before.

### 4.2. Cor, E, and NE Levels between Groups before and after Surgery

There is no significant difference in Cor, E, and NE expression levels between groups before surgery, and postoperative stress level increased in all groups, and G1<G2<G3<control group (*P* < 0.05), as shown in Table 5.

### 4.3. Intraoperative Anesthesia Time, Postoperative Eye Opening Time, and Extubation Time in Each Group

There are significant differences in intraoperative anesthesia time, postoperative eye opening time, and extubation time among all groups, anesthesia time and eye opening time G1>G2> G3>control group. However, the result of comparison of extubation time is G1< G2< G3<control group (*P* < 0.05), as shown in Table 6. The results show that the higher DEX dose is, the longer intraoperative anesthesia time and postoperative eye-opening time of patients will be. However, the extubation time is relatively shorter. It is further suggested that DEX has a highly selective excitatory effect on *α*2 adrenalin receptors in the locus coeruleus of the brain and can effectively inhibit the discharge function of neurons.

### 4.4. The Incidence of Postoperative Adverse Reactions

There are certain postoperative adverse reactions in all groups, and the total number of adverse reactions in G1 is significantly higher than that in other groups (*P* < 0.05), as shown in Table 7.

## 5. Conclusions

In this study, the effects of dexmedetomidine on hemodynamics and anesthesia effect of different doses of general anesthesia in patients undergoing hepatobiliary surgery are investigated. The experimental results demonstrate that during general anesthesia in the liver and gallbladder surgery, the patients with high dose of DEX can better maintain the intraoperative hemodynamic parameters and effectively restrain the postoperative stress reaction. However, they need a relatively long recovery time and will endure high probability of adverse events. Therefore, it is suggested to select different DEX according to the individual requirements and physical exertion of the patients in the process of clinical applications.

## Figures and Tables

**Figure 1:** Heart rate.

**Figure 2:** Systolic blood pressure.

**Figure 3:** Diastolic pressure.

**Table 1:** The baseline data.

Group	*n*	Age	Gender	
			Man	Woman
G1	24	36.64 ± 6.35	11(45.83%)	13(54.17%)
G2	24	35.98 ± 6.59	14(58.33%)	10(41.67%)
G3	24	36.07 ± 6.41	12(50.00%)	12(50.00%)
Control group	25	36.18 ± 6.53	10(40.00%)	15(60.00%)
*F/x * ^*2*^		2.267	5.623	
*P*		0.182	0.283	

**Table 2:** Changes of the heart rate in each group.

Group	*n*	T1	T2	T3	T4
G1	24	79.28 ± 3.02	80.56 ± 2.53	81.45 ± 3.42^a^	80.63 ± 3.29
G2	24	79.01 ± 3.21	80.30 ± 2.24	85.63 ± 3.52∗^ab^	81.24 ± 3.21∗^ac^
G3	24	79.18 ± 3.12	80.47 ± 2.35	88.35 ± 3.28∗^#ab^	82.42 ± 3.52∗^#ac^
Control group	25	79.21 ± 3.07	85.19 ± 2.38∗^a^	97.52 ± 6.63∗^#&ab^	86.73 ± 5.34∗^#&abc^
*F*		2.173	2.242	0.193	1.203
*P*		0.159	0.183	0.002	0.064

**Table 3:** Systolic blood pressure changes in each group.

Group	*n*	T1	T2	T3	T4
G1	24	119.32 ± 7.73	123.31 ± 7.83^a^	125.63 ± 6.45^a^	122.35 ± 6.72
G2	24	120.02 ± 7.39	123.75 ± 6.78	127.20 ± 6.85∗^ab^	123.04 ± 6.35^c^
G3	24	119.74 ± 7.29	122.67 ± 7.48	127.83 ± 7.52^ab^	123.46 ± 6.38^c^
Control group	25	119.92 ± 7.63	124.46 ± 6.83*∗*^a^	138.89 ± 8.42∗^#&ab^	125.62 ± 6.73∗^#&ac^
*F*		2.171	2.272	0.190	1.103
*P*		0.152	0.143	0.019	0.174

**Table 4:** Diastolic blood pressure changes in each group.

Group	*n*	T1	T2	T3	T4
G1	24	79.23 ± 5.89	80.32 ± 5.98	83.32 ± 5.62^ab^	80.02 ± 5.35^c^
G2	24	79.11 ± 5.21	80.73 ± 6.02	85.56 ± 6.02^ab^	81.36 ± 6.19^ac^
G3	24	79.28 ± 6.12	80.48 ± 5.74	86.78 ± 5.89^ab^∗^#^	81.63 ± 5.78^ac^
Control group	25	79.61 ± 5.07	80.34 ± 5.57	88.52 ± 6.42^ab^∗^#&^	82.22 ± 6.29^ac^
*F*		2.104	2.281	0.281	1.245
*P*		0.468	0.363	0.042	0.182

**Table 5:** Changes in stress levels in each group.

Group	*n*	Cor(mmol/L)		E(pmol/L)		NE(pmol/L)	
		Preoperative	Postoperation	Preoperative	Postoperation	Preoperative	Postoperation
G1	24	435.52 ± 10.21	674.32 ± 9.73	423.52 ± 9.85	643.22 ± 24.52	2455.26 ± 34.62	3213.44 ± 67.45
G2	24	432.46 ± 10.32	687.72 ± 10.02*∗*	425.63 ± 10.20	665.27 ± 23.45*∗*	2438.46 ± 36.42	3412.42 ± 67.83*∗*
G3	24	437.73 ± 10.25	698.42 ± 9.51*∗*^#^	424.46 ± 9.79	670.45 ± 25.32*∗*^#^	2431.35 ± 35.63	3534.45 ± 71.35*∗*^#^
Control group	25	436.73 ± 10.29	719.42 ± 10.52*∗*^#&^	426.24 ± 10.05	689.421 ± 27.52*∗*^#&^	2465.43 ± 36.35	3598.42 ± 71.39*∗*^#&^
*F*		1.234	4.353	1.246	5.325	1.194	5.624
*P*		0.192	<0.001	0.224	<0.001	0.172	<0.001

**Table 6:** Comparison of surgical indexes in each group.

Group	*n*	Anesthesia time(min)	Open time(min)	Extubation time(min)
G1	24	139.42 ± 20.22	39.46 ± 5.32	9.72 ± 4.23
G2	24	136.53 ± 20.19*∗*	36.45 ± 5.02*∗*	10.12 ± 4.28*∗*
G3	24	133.43 ± 20.26*∗*^#^	32.35 ± 4.87*∗*^#^	11.25 ± 4.19*∗*^#^
Control group	25	130.36 ± 19.39*∗*^#&^	27.35 ± 4.03*∗*^#&^	11.89 ± 4.29*∗*^#&^
*F*				
*P*				

**Table 7:** Adverse reaction comparison.

Group	*n*	Nausea	Vomiting	Respiratory depression	Restlessness	Total number
G1	24	3	**2**	4	4	13(54.17%)
G2	24	1	2	2	2	7(29.17%)
G3	24	2	1	1	2	6(25.00%)
Control group	25	1	1	0	2	4(16.00%)
*x * ^*2*^						5.342
*P*						<0.001

## Data Availability

The simulation experiment data used to support the findings of this study are available from the corresponding author upon request.
